# Evaluation and Analysis of Elderly Mental Health Based on Artificial Intelligence

**DOI:** 10.1155/2023/7077568

**Published:** 2023-02-09

**Authors:** Xiao Li

**Affiliations:** Faculty of Humanities and Social Sciences, Beijing University of Technology, Beijing 100124, China

## Abstract

**Objective:**

The purpose is to understand the depression status of the elderly in the community, explore its influencing factors, formulate a comprehensive psychological intervention plan according to the influencing factors, implement demonstration psychological intervention, and evaluate and feedback the effect, so as to provide a reference for improving the mental health of the elderly.

**Method:**

In order to make the output of different emotional data in LSTM more discriminative, a method to dynamically filter the output of LSTM is proposed. Combining the methods of Attention-LSTM, time-dimensional AI attention, and feature-dimensional AI attention, the best model in this paper is obtained. The multistage stratified cluster sampling method was used to conduct a questionnaire survey on the elderly aged 60 and above in a certain area, including the general demographic characteristics questionnaire of the elderly, the self-rating scale of mental health symptoms, and the health self-management ability of adults. All data were entered into a database using Excel software, and SPSS 19.0 statistical software was used for statistical analysis. *Results/Discussion*. The detection rate of depression (GDS ≥ 11 points) among the elderly in a community in a certain area was 39.38%. Multivariate logistic regression analysis showed that family history of mental illness, more negative life events, decreased ability of daily living, living alone, and suffering from physical diseases in the past six months were the risk factors for depression in the elderly. Community health education can partially alleviate depression in the elderly. The detection rate and degree of depression of the elderly in the comprehensive psychological intervention group were significantly lower than those in the control group, and the difference was statistically significant (*P* < 0.05).

## 1. Introduction

The 21st century will be a century of population aging, and the aging of countries in the world is rapidly attacking, which is characterized by a large number, a high speed, and a large proportion of the elderly [1]. The period from 2001 to 2020 is a period of rapid aging in China. By the end of 2020, the proportion of China's elderly population aged 60 and above has reached 14.9% of the total population, or about 202.43 million people. Among them, the population aged 65 and above has reached the total population [2]. The proportion of the population is 9.7%, and the number is still increasing by more than 8 million every year. The aging of the population is becoming more and more serious, which brings severe challenges to society, economy, and medical care [3]. In addition, with the continuous development of social economy, people are more and more aware of the importance of health, and medical and health resources can no longer fully meet the health needs of the elderly. As a new medical care model, health self-management has attracted great attention, which is of great significance to improving the quality of life of the elderly and promoting healthy aging [4].

If the elderly cannot properly deal with these problems, it is easy to have bad psychological states such as depression, loneliness, anxiety, despair, and fear, which will not only bring pain and misfortune to the elderly themselves but also increase the burden of disease on the family and society [5]. Therefore, researching and paying attention to the mental health status of the elderly and strengthening the psychological protection of the elderly are one of the important contents of the elderly's health care undertaking and one of the priorities of community services [6].

As the public is influenced by the traditional concept of “emphasizing the body and ignoring the mind,” many elderly people take an ignoring attitude towards their own psychological problems and seldom actively seek mental health services, so that many suffer from depression or mild depression [7]. The elderly in the community cannot get timely intervention, which leads to the chronic persistence of mental illness and causes depression [8]. Therefore, understanding the epidemiological status and influencing factors of depression among the elderly in the community, early identification and early intervention have huge economic and social benefits [2, 9, 10].

This paper first introduces the traditional LSTM output and focuses on the use of the LSTM output in the voice mental health assessment task for the elderly. Subsequently, this paper proposes two improved LSTM output methods: automatic screening using artificial intelligence attention in time dimension or artificial intelligence attention algorithm in feature dimension. Then, this paper fuses the artificial intelligence attention algorithms in the time dimension and feature dimension and fuses the successfully fused model with Attention-LSTM; that is, the fusion of the three artificial intelligence attention models is completed, and the result in this paper is obtained.

This research is the first time to conduct a large-scale survey on the mental health of the elderly in a certain area, especially to research and analyze the chronic diseases of the elderly closely related to the mental health of the elderly, economic and pension security, and support systems, and actively seek to influence the elderly. It is very urgent and important to improve the mental health of the elderly, which is conducive to promoting the construction of active and healthy aging in a certain area, and has far-reaching significance for building a harmonious society.

Depression is common among the elderly in the community in a certain area, and the level of depression is relatively high; the occurrence of depression in the elderly in the community is mainly affected by family history of mental illness, daily living ability, living style, physical illness and life events in the past six months, social support, etc. Comprehensive psychological intervention can effectively improve the depression of the elderly in the community.

## 2. Methods

### 2.1. LSTM Output Method in Elderly Mental Health Assessment Task

LSTM is usually used to model temporal information, such as speech, text, or images with temporal relationships (such as video). Typically, there are two registers inside an LSTM, the “hidden layer output” and the “cell state.” For temporal input features, the LSTM has a set of outputs corresponding to the input of each frame. In speech enhancement tasks, it is usually necessary to use the hidden layer output of each frame for regression tasks, such as reconstructing the power spectrum of this frame or floating-value concealment.

In the task of speaker identification, it is necessary to extract an embedding from the output of LSTM, such as extracting X-vector and pooling of sequential coding, and then calculate the distance or cosine similarity between this embedding and a specific speaker. In speech emotion recognition task, we typically think it includes all valid information in the process of recursion and then enter the subsequent full connection layer and layer softmax emotion classification.

Many scholars have conducted research on how to improve the output of traditional LSTM. The LSTM described above picks the last moment as the output [2, 6]. This may result in the LSTM output information at other historical moments not being fully utilized. Specifically, since the time span of long-term dependencies is not infinite, the accumulated information of the last-minute LSTM is actually lossy.

This section takes the last output as baseline to ensure that it can gain a larger weight by using the AI attention mechanism. In addition, considering the difference of discrimination ability between speech features, this section proposes the AI attention algorithm of time dimension and the AI attention algorithm of feature dimension and compares it with baseline.

### 2.2. AI Attention in Time Dimension

1. Although hT contains the historical information of each previous moment, it does not necessarily contain useful information. For example, in the LSTM recursive process, the information that is more obvious to the emotional category in a certain frame may be assigned by the forget gate.
2. In the input speech sentence (utterance), there may be a large number of silent frames or noise-containing segments, and these parts contain very little emotional information
3. In speech containing emotion (especially in natural emotion corpus and guided emotion corpus), the transformation of emotion usually has a progressive relationship, and the artificial intelligence attention algorithm on the output of the time series can help improve the recognition rate of emotions

Since the degree of emotional information contained in different frames is not uniform, it means that the contribution of these frames to the emotion recognition of the final model is different; that is to say, the degree of these contributions can be represented by the weight coefficient of the frame. The authors calculate the weight coefficients based on the output of the encoder and the current input of the decoder based on the artificial intelligence attention mechanism and then weight the output of the encoder for use by the input of the decoder at the next moment. The local AI attention mechanism is used to calculate the weights of different frames with the AI attention parameter vector as described in the following equation.

(1) $$\begin{array}{c} \alpha_{t}=\exp\left(y_{t}u_{H}\right)•\overset{T-1}{\underset{i=0}{\prod }}\exp{\left(y_{i+1}u_{H}-y_{i}u_{H}\right)}^{-1}, \end{array}$$

where exp is the exponential operation and *T* is the total number of frames of the current utterance.

Considering the artificial intelligence attention weighting of the time dimension on the output of LSTM, through the recursive memory module of LSTM, the LSTM output at the last moment actually contains the most historical information. Therefore, the last-minute LSTM output should be weighted the most. This section uses the last-minute output as a reference to use the cosine similarity to calculate the weight of the output at all times to ensure that it can get a larger weight through the attention mechanism (the cosine similarity calculated by itself and itself gets the largest weight). Finally, the weight coefficients are applied to the output of the full LSTM and summed over the time dimension as the output. The relevant calculation formula is

(2) $$\begin{array}{c} s_{T}=\text{softmax}\left[{\left(w_{t}•x_{T}\right)}^{H}•x_{T-1}\right],\\ \text{outpu}{\text{t}}_{T}=\left(1-s_{T}\right)•x_{T-1},\\ H\left(x\right)=\left(1-W_{a_{F}}\right)F\left(-x\right)-2x•W_{a_{F}}. \end{array}$$

### 2.3. AI Attention in Feature Dimension

It is well known that it is difficult to use a single feature to complete multiclass classification tasks, so it is often necessary to combine multidimensional features to complete these classification tasks. However, the features of each dimension are not the same as the distinguishability of the target task. The features of the elderly mental health assessment corresponding to different dimensions are easier to be identified by the model.

In speech emotion recognition tasks, the last output of the above LSTM (which can be the traditional last minute output, or the output after the artificial intelligence attention screening in the temporal dimension proposed in this section) is usually directly sent to the fully connected layer and then sent to the softmax layer for classification.

If the initialization method of parameters in the fully connected layer is a standard normal distribution with mean 0 and variance 1, it can be regarded as fair treatment for all LSTM outputs (regarded as coding features of utterance).

In order to express the differences between features, this section proposes a self-AI attention calculation method on feature dimensions to calculate the AI attention weight of features of different dimensions, so as to automatically screen out the discriminative emotional features from the output of LSTM and send them to the subsequent fully connected layer for classification.

To express the difference between features, the AI attention weights are calculated on the feature dimension as follows:

(3) $$\begin{array}{c} s_{F}=\text{softmax}\left[\cot h\left(v_{F}-w_{F}\right)•x_{T-1}\right],\\ \text{outpu}{\text{t}}_{F}=\underset{\text{time}}{\prod }\left(1-x_{T-1}\right)•s_{F-1}. \end{array}$$

The input dimension of these two matrices is *N*, and the output dimension is also *N*. It indicates that the corresponding elements are multiplied, that is, the dot multiplication operation.

The summation is carried out on the time dimension, and its purpose is to compute the statistical function of the characteristics on the time dimension. Note that the mean operation can also be used here, but the actual number of frames for different samples is not consistent (i.e., the padding effect on short utterance should be considered). Similarly, here, [*B*, *N*] represents the number of hidden layer units of batch size and LSTM.

### 2.4. Fusion Attention-LSTM, Time Dimension AI Attention, and Feature Dimension AI Attention

This section fuses Attention-LSTM with AI attention in time dimension and AI attention in feature dimension. These three artificial intelligence attention algorithms can be regarded as three modular algorithms proposed for speech emotion recognition; that is, they can individually improve the performance of emotion recognition and optimize the time complexity of training. And the three modules are fully integrated together. The first is the fusion of the artificial intelligence attention algorithm in the time dimension and the artificial intelligence attention algorithm in the feature dimension. This paper tries three fusion methods:

1. First, do the time dimension artificial intelligence attention to filter the time dimension, and then perform the feature dimension artificial intelligence attention algorithm on the filtered features to filter the feature dimension
2. Perform feature dimension AI attention to filter the feature dimension, and then perform the time dimension AI attention algorithm on the filtered features to filter the time dimension
3. Simultaneously and in parallel, filter the time dimension and feature dimension of the output of the LSTM, and then fuse (splicing or adding) the two filtered features

Integrating Attention-LSTM, time dimension AI attention, and feature dimension AI attention algorithm framework is shown in Figure 1.

In the research process of fusion algorithm, it is found that the first two methods will lead to the model that can not be trained, and the performance of recognition rate will always fall into a small shock near the extreme point.

Attention after analysis, this paper argues that a variety of artificial intelligence algorithm will “serial” serious cause before to the spread of the value is too small (especially in the attention to training parameters of the algorithm of artificial intelligence is still in the random initialization phase and will be serious damage to the spread of information) and will cause serious gradient back propagation problems disappear.

Usually, the solution to this problem is to use a residual structure. The splicing of method 3 significantly improves the performance of emotion recognition and is better than the addition method. The analysis in this paper holds that the order of magnitude of the output parameters of the two AI attention modules may not be the same (for example, some of them may be negative), and simple addition is equivalent to weighting the two modules to 1, respectively.

However, the order of magnitude of these features can not represent their importance in the subsequent network, nor can it prove that the importance of the two AI attention modules is the same, so the splicing method is significantly better than the addition method.

### 2.5. Research Objects

#### 2.5.1. Sample Size Calculation

The sample size of this survey is determined by the following formula: *N* = 400*Q*/*P*, where *P* in the formula is the two-week prevalence rate of the elderly. According to the presurvey results, the two-week prevalence rate of the elderly in the community is 34.0%.

#### 2.5.2. Selection of Research Subjects

The subjects of the study were elderly residents aged 60 and over in 3 districts of a region.

1. Inclusion criteria of research subjects: those who have formal household registration in the three regions selected in a certain region and have lived in the survey site for one year or more, as of the time of the survey, are ≥60 years old
2. Exclusion criteria for study subjects:

- Severe illness, mental illness, senile dementia, and severe cognitive impairment
- Due to various reasons, the expression is unclear and the communication is impaired
- Those who refuse the survey and those who go out to live during the survey

### 2.6. Sampling Method

This study adopts the method of multistage stratified cluster sampling and selects 3 areas in a certain area as sample areas. The first stage takes the city as the sample area; the second stage takes the urban area (county) as the sample area; the third stage takes the street (township) as the sample area; the fourth stage takes the community (village) as the sample area.

The research objects were selected in cities and rural areas, and one urban area and one county were randomly selected in each of the three cities using the digital lottery method. The cluster selects communities and natural villages in the jurisdiction and conducts a questionnaire survey on all eligible research subjects. A questionnaire survey was conducted on the elderly who met the inclusion and exclusion criteria in the selected communities and natural villages. The effective recovery rate of this survey was 98.19%.

### 2.7. Quantitative Research

This study mainly used questionnaires to collect data. The research tools included six questionnaires: questionnaires on general demographic characteristics of the elderly, self-assessment scale for symptoms, assessment scale for adult health self-management ability, family function assessment scale, Social Support Rating Scale, and Daily Living Ability Scale.

#### 2.7.1. General Demographic Characteristics Questionnaire

The general demographic characteristics questionnaire was designed by the researchers, mainly including the elderly's residence, gender, age, marital status, education level, economic status, medical and pension insurance, physical discomfort, care for children and family members, and chronic diseases. The diagnostic criteria for chronic diseases include (1) those who have been diagnosed with chronic diseases by hospitals at or above the county level within six months of the investigation and (2) those who have been diagnosed with chronic diseases by hospitals at or above the county level six months ago which have frequent attacks during six months of the investigation and have responded accordingly.

#### 2.7.2. Assessment Tool for Adults' Health Self-Management Ability

The adult health self-management skill assessment scale (AHSMSRS) has 38 items in three dimensions: self-management behavior (14 items), self-management environment (10 items), and self-management cognition (14 items). Using likert 5-level scoring method, the evaluation standards of each subscale are different. Health self-management cognition subscale using “agree, somewhat agree, uncertain, less agree, disagree” and “confident, more confident, uncertain, less confident, no confidence”. The total score range is 38-190 points, with a total score of 38-76 as low-level support, 77-152 as medium-level support, and 153-190 as high-level support. The higher the total score, the higher the level of healthy self-management.

#### 2.7.3. Family Function Rating Scale

The lower the score of each dimension, the better the corresponding family function. The total score is 60-240 points, and the family function is divided into three sections according to the score. 60-120 points indicate good family function, 120-180 points indicate average family function, and 180-240 points indicate poor family function.

### 2.8. Data Collection

In the field investigation, in order to improve the compliance of the subjects, the investigators provided free physical examination and small gifts for the elderly with self-provided instruments such as blood pressure monitor, electrocardiogram machine, and bone density meter. Questionnaires were handed out on the spot during the survey. After the investigators explained the purpose with unified instructions, the questionnaires were generally handed out to the elderly and asked to fill in by themselves. If the elderly had difficulties in filling in, the investigators read out each question for them and gave detailed explanations to the items that had difficulties in understanding. After filling in the questionnaire, the investigators should check it in time. If there is any doubt, they should inquire and correct it in time.

#### 2.8.1. Questionnaire Design Stage

Check the literature, compile the questionnaire according to the research content, ask the relevant experts to review the self-designed questionnaire after the compilation, and conduct a preinvestigation to test the rationality and feasibility of the questionnaire, and repeat and supplement the questionnaire to ensure the investigation.

#### 2.8.2. Investigators

Through formal training, each investigator is required to clarify the purpose of the investigation, be familiar with the contents of the questionnaire, master the methods of investigation and inquiry, measure methods, etc., to ensure that the measurement is accurate.

#### 2.8.3. On-Site Investigation

Investigators should follow the ethical principle of informed consent before conducting investigations, brief the respondents on the research content and procedures, the identity of the investigators, ensure that the investigation is harmless, and follow the principle of confidentiality to keep the information of the respondents absolutely confidential. After each questionnaire is completed, the investigators should check it in time. If there is any doubt, they should ask and correct it in time. If any omission is found, it should be filled in time, so as to ensure the qualification and scientificity of the questionnaire as much as possible. Immediately, some respondents (5%) were selected for reexamination, and the two results of the same batch of respondents were compared to evaluate the quality of the survey.

#### 2.8.4. Data Quality Control

After the on-site investigation, the questionnaires were sorted out, and the questionnaires with unfilled items exceeding 20% of the entire questionnaire were eliminated; the questionnaire items were sorted and coded, and the data entry personnel were trained uniformly to ensure the consistency of data entry; after the data entry was completed, check the logical error; if there is a problem, check with the original questionnaire in time to ensure the authenticity of data entry.

#### 2.8.5. Statistical Analysis

All data were entered into a database using Excel software, and SPSS 19.0 statistical software was used for statistical analysis. Measurement data were expressed as *x* ± *s*, *t*-test and variance analysis were used for univariate analysis, and multiple stepwise regression analysis was used for multivariate analysis.

Semistructured interview is adopted in this study, through which the elderly can have a more direct understanding of the subjective understanding, position, and emotion of an event and an object, so as to conduct a comprehensive summary and analysis of their mental health status and behavior. The interview method is an in-depth survey, a supplement and extension of the questionnaire method.

## 3. Results

### 3.1. Quality Evaluation of Data

There was no significant difference in the composition of general data such as gender, age, household registration, and residence style between the lost-to-follow-up group and the surveyed group (*P* > 0.05). The age distribution of the elderly in the lost-to-follow-up group and the response group is shown in Figure 2. The general demographic data of the elderly in the community are shown in Table 1.

Among the elderly in the community, 34.8% reported that they had suffered from physical diseases in the past six months, and 65.2% reported no new physical diseases; 5.18% reported that they had a family history of mental illness, and 94.82% reported no family history of mental illness (see details in Table 2).

The total score of the SSRS scale and the three dimensions of the social support scale for the elderly in the community are total social support score (28.78 ± 6.89), objective support (4.71 ± 2.38), and subjective support (18.32 ± 4.27).

### 3.2. Activities of Daily Living

The total score of the community elderly ADL scale was between 13.00 and 5.00, with a median of 16.00 and an interquartile range of 7.00. Physical self-care skill (PSMS) subscale scores ranged from 6.0 to 24.00, with a median of 7.00 and an interquartile range of 1.00. The instrumental activities of daily living (IADL) subscale scores ranged from 7.00 to 33.00, with a median of 11.00 and an interquartile range of 7.00.

According to the standard of ≥2 items with a score of ≥3 or a total scale score of ≥22, a total of 233 (16.8%) elderly people in this survey had varying degrees of functional decline; 1156 had normal activities of daily living (≤20 points), accounting for 83.2%. The activities of daily living (ADL) of the elderly in the community are shown in Figure 3.

### 3.3. Univariate Analysis

The *χ*^2^ test was used to compare the effects of different factors on the occurrence of depression among the elderly in the community. The results showed that factors such as age, family economic status, family history of mental illness, life events, social support, marital status, cognitive function, physical health status in the past six months, and activities of daily living and living with others were all associated with depression among the elderly in the community. The single factor effect of depression is shown in Figure 4.

### 3.4. Multivariate Analysis

Taking the presence or absence of depression as the dichotomous dependent variable (GDS < 11 points = 0 and GDS ≥ 11 points = 1), multivariate logistic regression analysis was performed on elderly people in the community. They were gradually included in order, and the inclusion criterion was *P* = 0.05, and the exclusion criterion was *P* = 0.10.

The results showed that six factors including ADL (X5), LES (X8), SRSS (X9), living style (X3), physical health status in the past six months (X6), and family history of mental illness (X2) finally entered the regression equation. The combined equation was statistically significant (*χ*^2^ = 107.834, *P* = 0.001). Family history of mental illness, decreased ability of daily living, living alone, physical illness, and major life events in the past six months are risk factors for depressive symptoms in the elderly, and good social support is a protective factor for depression in the elderly, as shown in Table 3.

### 3.5. The Effect of Different Intervention Programs on the Degree of Depression among the Elderly in the Community

There were 50 people in both groups at the time of enrollment. After the intervention, there were 47 remaining cases in the control group, and 3 were dropped out, with a loss-to-follow-up rate of 6.00%. Among them, 2 were lost to follow-up due to illness and hospitalization, and 1 dropped out due to going out to visit their children. There were 46 remaining cases in the intervention group, 4 of whom dropped out, and 2 of them dropped out. One was lost to follow-up due to illness, one was dropped out due to lack of time to take care of his wife, and one died unexpectedly, with a loss-to-follow-up rate of 8.00%. The final sample size of this study was as follows: the control group (*n* = 46) and the intervention group (*n* = 47), a total of 93 people; the total loss to follow-up rate was 7.00%, and the loss to follow-up did not affect the results. The equilibrium test showed that there were no significant differences in general demographic data and GDS scores between the two groups before the intervention (*P* > 0.05), and the two groups were comparable. The specific data are shown in Table 4.

Paired group *t*-test was used for intragroup comparison. The results showed that the GDS score of the elderly in the control group was significantly reduced after general health education, and the difference was statistically significant (*P* = 0.046). The elderly in the intervention group received general health education combined with comprehensive psychological intervention. Before the GDS score was significantly lower than the baseline value, the difference was statistically significant (*P* = 0.001).

The independent sample *t*-test was used to compare the groups, and the results showed that there was no significant difference in the GDS scores of the elderly in the two groups before the intervention (*P* = 0.91); after the 3-month intervention, the score was lower than that of the elderly in the control group, and the difference was statistically significant (*P* = 0.002).  Figure 5 shows the comparison of the GDS scale scores of the depression level before and after psychological intervention for the elderly in the community in the two groups.

## 4. Discussion

### 4.1. Strategies and Methods for the Preparation of Mental Health Scales for the Elderly in a Certain Area

Mental health scale preparation strategies can be roughly divided into three methods: rational-theoretical strategy, factor analysis strategy, and criterion control strategy [11–13]. Among them, the rational-theoretical strategy requires the compiler to compile the scale according to their own theories or assumptions, such as the Edwards Personal Preference Scale (EPPS). Class or factor analysis method is a method of scale preparation, such as the Cartel Sixteen Personality Questionnaire and the Eysenck Personality Questionnaire; the criterion control strategy pays more attention to the validity of the compiled items and scales, such as Minnesota Polyphasic Personality Inventory [14]. In fact, in the process of compiling the mental health scale, researchers are not limited to one method but more comprehensively use various methods, that is, apply comprehensive strategies to compile [15].

### 4.2. Discussion on the Reliability and Validity of the Mental Health of the Elderly in a Certain Area

In this study, two indicators are proposed to test the reliability of the questionnaire, namely, the internal consistency reliability, namely, Cronbach's alpha coefficient, and the split-half reliability [16]. After statistical analysis, the overall internal consistency coefficient of the questionnaire was 0.924, and the internal consistency coefficient of each dimension was between 0.626 and 0.962. The split-half reliability of the total questionnaire is 0.658, and the split-half reliability of each dimension is between 0.584 and 0.950, which makes the reliability index of the questionnaire relatively ideal, with better reliability and stability [17].

In the process of preparation, relevant professionals and graduate students of this major (see above) were invited to evaluate and modify the questionnaire items and the expression of items, so as to make the meaning of the items clearer. Then, some elderly subjects were invited to read and evaluate the questionnaire to make it more consistent with the reading preferences of the elderly. After further modification of the questionnaire, a formal questionnaire on the mental health of the elderly in a certain area was finally formed, so the content validity of this questionnaire was also good.

After exploratory factor analysis in this project, the five-factor structure of the questionnaire was obtained, and the researcher conducted a confirmatory factor analysis on the questionnaire [18]. The analysis results showed that the questionnaire structure fits well. The correlations between the questionnaires are relatively significant, and the correlation coefficient between the items and the total score is between 0.299 and 0.692, indicating that the correlation coefficient is significant; the correlation coefficient between the scores of each subdimension of the questionnaire and the total questionnaire score is 0.383. Between -0.775, all are at a significant level, which effectively indicates that the overall concept of the total questionnaire has a strong consistency with each dimension, and it shows that the questionnaire structure has a strong rationality [19].

In the formal testing process of this study, in addition to requiring the subjects to complete 45 items, an additional item to measure the validity of the criterion was added, namely, “46. I am mentally healthy” [20]. The results showed that, in addition to the “cognitive efficacy” dimension, the calibration scale had a significant correlation with the other four subdimensions and the total score. Among them, the school standard was significantly negatively correlated with “suspiciousness and denial,” indicating that if the elderly feel that they are mentally healthy, they will have less negative emotional experience, which is in line with theoretical expectations [17, 21, 22].

### 4.3. Discussion on the Mental Health of the Elderly in a Certain Area

The results of this study show that males are significantly lower than females in terms of happiness score, and males are significantly higher than females in terms of cognitive efficacy [23–25]. Although there is no significant difference in the total score of happiness, from these two important dimensions, among the elderly in Chongqing, male cognitive performance is better, while female is happier [26]. This is consistent with social and cultural standards. Men are more engaged in outside work and pay attention to matters at the national level, so their cognitive functions age more slowly, while women pay more attention to family, children, and grandchildren linger, and women's spare time life is more colorful, making them feel happier. Age has an important impact on the happiness of the elderly in Chongqing. With the increase of age, the happiness score shows a significant downward trend. This reminds us that with the decline of bodily functions, the older we get, the more care and attention we need from our family and society [27–29].

On the contrary, happiness increases with the level of education. On the one hand, people with different levels of education have different views on the meaning of life and death [30]. Interestingly, happiness is not directly proportional to wealth. The elderly with average economy and high level are happier than the very poor and very rich [18, 31]. The former occupation is an agency, and the happiness of the elderly in the enterprise is significantly higher than that in other occupations [32–34].

Judging from the current results on the mental health of the elderly in a certain area, we need to strengthen the care for the elderly. According to different groups and components, different policies and systems need to be formulated to improve the mental health of the elderly.

### 4.4. Reflections on the Three No Elderly Groups in Welfare Homes

The elderly, as a special group that cannot be ignored, in the last stage of their life course, we generally believe that what they lack and need most is the company and communication of their families [35]. As one of the vulnerable groups in society, the state has placed the elderly in the welfare home for assistance in order to make their lives convenient and worry-free and provided free accommodation, food, and various daily necessities for the elderly through fund allocation [36]. The Sanwu elderly living in the orphanage can already be satisfied in terms of material [37]. In the conversation between the researcher and the elderly Sanwu, the elderly Sanwu also expressed their material satisfaction to the researcher. However, there are serious deficiencies in the mental and social aspects of the elderly in the welfare home [24, 38, 39].

What are the real needs of the Sanwu elderly in the welfare home? What can be done to allow the elderly in the hospital to enjoy their old age? This is something we need to consider and reflect on. Social work believes that everyone has the right to survive and develop. We cannot deprive the development rights of the elderly in the hospital.

### 4.5. Reflections on Social Support Theory

Under the guidance of social support theory, this research is relatively successful. As a universal social phenomenon, social support is essential for everyone in daily life. Insufficient social support often leads to personal distress [40–42]. Social support theory believes that individuals or families are in trouble because their social support network is “broken” [43, 44]. Support network, community support network, national support network, and social support network are analyzed to provide the basis for social work intervention [45–47].

Under the guidance of social support theory, workers often appear as “reconstructors” of social support networks. It is oriented to the needs of the clients, with material support, emotional support, and information support as the mediator, to help the clients establish an effective social support network. This can not only meet their current needs and help the client get out of the predicament and return to a normal life but also help the client form a long-term effective communication mechanism, make the client return to a normal life, and help the client achieve good social integration.

The traditional social support theory analyzes the family support network, community support network, national support network, and social support network to carry out activities for the three-no-elderly elderly [35, 48]. However, it is difficult to find the particularity of the group and its fundamental needs if it is still analyzed from the perspective of the traditional social support theory for a special group such as the elderly with three nos [49].

In the face of this situation, social support theory should combine with the local reality of China in the process of the change of discourse system and knowledge structure and adhere to the cultural sensitivity of professional social work practice and the inevitability of social work practice in different situations.

## 5. Conclusion

This paper proposes two improved LSTM output methods: automatic screening by using the time-dimension AI attention or the feature-dimension AI attention algorithm. Then, this paper fuses the artificial intelligence attention algorithms of the time dimension and feature dimension and fuses the successfully fused model with the Attention-LSTM proposed in the previous point; that is, the fusion of the three artificial intelligence attention models is completed. The detection rate of depression among the elderly in a community in a certain area was 39.38%, and the GDS score of depression level was 10.52. Univariate *χ*^2^ analysis showed that there were nine factors including age, family economic status, family history of mental illness, life events, social support, cognitive function, marital status, physical health status in the past six months, and ability of daily living and living with others. Multivariate logistic regression analysis showed that family history of mental illness, decreased ability of daily living, more negative life events, physical illness in the past six months, and living alone were the main causes of depression in the elderly. The depression level of the elderly in the community in a certain area is higher than that of the normal population. The incidence of depressive symptoms in the elderly in a certain area is higher than that in the normal population. Family history of mental illness, living alone, suffering from physical disease in the past six months, more negative life events, and decreased ability of daily living are risk factors for depression in the elderly; good social support is a protective factor for depression in the elderly. Implementing health education in the community can help alleviate depression in older adults. The effect of implementing comprehensive psychological intervention combined with health education in the community is better than that of simple health education, and the degree of depression and the detection rate of the elderly are significantly reduced.

## Figures and Tables

**Figure 1:** Integrating Attention-LSTM, time dimension AI attention, and feature dimension AI attention algorithm framework.

**Figure 2:** The age distribution of the elderly in the lost-to-follow-up group and the response group.

**Figure 3:** Activities of daily living (ADL) of the elderly in the community.

**Figure 4:** Univariate analysis of depression.

**Figure 5:** Comparison of GDS scale scores of depression level before and after psychological intervention for the elderly in the community.

**Table 1:** General demographic data of the elderly in the community.

Indicator	Classification	Composition ratio (%)
Way of living	Living alone	84.6
	Not living alone	15.4
Marital status	Unmarried	6.1
	Married	73.4
	Divorced	1.9
	Remarry	8.6
	Widowed	10
Nationality	Han nationality	92.7
	Minority	7.3
Household registration	Town	10.9
	Rural	89.1
Gender	Male	52.2
	Female	47.8

**Table 2:** Physical diseases of the elderly in the community in the past six months.

Indicator	Physical illness		Family history of mental illness	
Classification	Y	N	Y	N
Composition ratio (%)	33.6	66.4	2.7	97.3

**Table 3:** Multivariate logistic regression analysis of depression among the elderly in the community.

	Physical illness in the past six months	Have a family history of mental illness	More negative life events	Decreased ability of daily living	Living alone	Good social support	General social support
OR	1.2	1.0	0.8	1.3	0.6	1.5	0.65
Wald	4.6	6.3	5.2	8.1	4.7	10.5	9.4
95% CI	1.4	0.7	0.9	0.6	1.2	1.3	1.1
SE	0.11	0.14	0.13	0.12	0.15	0.13	0.17
Sig.	0.01	0	0	0.02	0	0	0.01

**Table 4:** Comparative analysis of the general data of the elderly in the two groups of community.

Indicator	Classification	Control group	Intervention group
Way of living	Living alone	36	31
	Not living alone	24	29
Marital status	Unmarried	3	5
	Married	30	32
	Divorced	7	6
	Remarry	12	10
	Widowed	8	7
Nationality	Han nationality	53	56
	Minority	7	4
Household registration	Town	9	10
	Rural	51	50
Gender	Male	35	36
	Female	25	24

## Data Availability

The data used to support the findings of this study are available from the corresponding author upon request.
